The article "A Reliable Machine Intelligence Model for Accurate Identification of Cardiovascular Diseases Using Ensemble Techniques" was published in 2022. Journal: J Healthc Eng.

# A Reliable Machine Intelligence Model for Accurate Identification of Cardiovascular Diseases Using Ensemble Techniques

**DOI:** 10.1155/2022/2585235

**Published:** 2022-03-08

**Authors:** Bhanu Prakash Doppala, Debnath Bhattacharyya, Midhunchakkaravarthy Janarthanan, Namkyun Baik

**Affiliations:** ^1^Department of Computer Science and Multimedia, Lincoln University College, Kuala Lumpur 47301, Malaysia; ^2^Computer Science and Engineering Department, Koneru Lakshmaiah Education Foundation, Vaddeswaram, Guntur 522302, India; ^3^Busan University of Foreign Studies, Geumjeong-gu, Busan, Republic of Korea

## Abstract

Machine intelligence can convert raw clinical data into an informational source that helps make decisions and predictions. As a result, cardiovascular diseases are more likely to be addressed as early as possible before affecting the lifespan. Artificial intelligence has taken research on disease diagnosis and identification to another level. Despite several methods and models coming into existence, there is a possibility of improving the classification or forecast accuracy. By selecting the connected combination of models and features, we can improve accuracy. To achieve a better solution, we have proposed a reliable ensemble model in this paper. The proposed model produced results of 96.75% on the cardiovascular disease dataset obtained from the Mendeley Data Center, 93.39% on the comprehensive dataset collected from IEEE DataPort, and 88.24% on data collected from the Cleveland dataset. With this proposed model, we can achieve the safety and health security of an individual.

## 1. Introduction

Cardiovascular disease (CVD) is considered a prevalent and dangerous human ailment in recent days. According to the World Health Organization (WHO), more than 40 million deaths caused in the last decade due to noncommunicable diseases; one among them is CVD. One-third of these deaths occurred in the countries that fall under low-income and middle-income groups. According to the statistics provided by the Centers for Disease Control and Prevention (CDC), in America, one in every four deaths is caused due to heart diseases, which is about 610,000 deaths per year. Many factors such as high blood pressure, excessive alcohol consumption, cholesterol, stress, and obesity are playing a pivotal role.

Different types of CVDs are as follows: angina which is mainly caused due to decreased blood flow into the heart, arrhythmia caused by an irregular heartbeat, a faster heartbeat can be considered as tachycardia, and a slower one can be considered as bradycardia, congenital heart disease is an issue that occurs due to the heart's anatomy at the time of birth [1], heart disease that affects the arteries can be considered as coronary artery disease, sudden blockage of blood and oxygen flow can be treated as an heart attack, and if the condition affects the contrast and relaxation of the heart, it can be considered as heart failure. Based on the disease type, proper diagnosis and treatment are required to avoid the worst conditions. Heart infections may be caused by different viruses, parasites, or any kind of hazardous bacteria. Atherosclerosis is a circumstance that develops a substance known as plaque which builds up in artery walls. Because of this, heart arteries will become narrow, and blood flow will be tough to pass through, leading to stroke. The first kind is ischemic stroke (the maximum common form of stroke); when it occurs, blood vessels will be blocked, which is typically a form of a blood clot. When blood vessels inside the brain burst out, it is identified as hemorrhagic stroke that is caused due to hypertension (high blood pressure). Stenosis occurs if coronary heart valves do not open sufficiently and block blood from flowing through them freely. Early diagnosis of the diseases with precise medical tests can increase the chances of survival and saves time. Healthcare professionals are rigorously working in this area for many years to help humankind. Based on a survey, it is stated that CVD is the leading cause to several deaths in the United States of America [2].

The article "A Reliable Machine Intelligence Model for Accurate Identification of Cardiovascular Diseases Using Ensemble Techniques" was published in 2022. Journal: J Healthc Eng.

Artificial intelligence (AI) plays a prominent role in making better medical condition analysis and diagnosis decisions in the healthcare industry. It is also known as deep medicine, which has enough capability to acquire data and can produce a well-defined output by processing them [3].

Several research studies and articles state that AI can outperform healthcare-related tasks better than humans. Machine learning (ML) and deep learning (DL) algorithms are being employed in different kinds of disease classification and identification purposes [4]. ML can be considered to be a statistical technique in fitting data to models. The process of training enormous kinds of data to the model can lead to unleashing better accuracy. According to the survey conducted by Deloitte in 2018, managers in the USA stated that companies already incorporated AI techniques up to 63% in their respective business models. In the healthcare industry since 1970, these models perform more specific tasks such as disease prediction and detection. For example, for identifying blood-borne infections related to bacteria, MYCIN was made at Stanford University [5]. In recent findings, IBM's Watson focused on prescribing exact medicine, especially for diagnosing cancer, and helped to provide exact treatment. TensorFlow from Google's invention also helped researchers to develop different kinds of applications.

The article "A Reliable Machine Intelligence Model for Accurate Identification of Cardiovascular Diseases Using Ensemble Techniques" was published in 2022. Journal: J Healthc Eng.

Medical facilitators and service providers use their clinical expertise to develop different plans to take care of and improve patients' health from different chronic health conditions. General suggestions are always advisable, such as losing excess weight, doing regular workouts, and keeping track of continuous clinic visits based on the patients' health condition. However, significant problems occur when a patient does not follow the prescribed treatment [6].

One of the shortfalls noticed during these days was the transparency of the technology. Most AI models, especially DL algorithms, mainly focus on analyzing the image, which are impossible to explain virtually. In most cases, patients will try to know their disease and its stages. Medically, it is possible to explain the symptoms and disease identifications to a patient, but through these DL techniques, it is complicated [7].

We believe AI can play a vital role in the healthcare industry with ML and DL algorithms. It is capable of providing the best precision values towards disease identification and diagnosis. Medical practitioners must include technologies in their daily medical practices to develop better systems to help humankind.

Making the right decision at a low price is essential and helpful for health experts and patients with better treatment. It is possible by creating an intelligent system to minimize the damage. Besides, the known fact is that technology is not made available everywhere [8]. In this study, a reliable ensemble model has been proposed which identifies the disease with better accuracy.

## 2. Related Work

AI-Milli [9] preferred an associate strategy for CVD classification using neural network (NN) variation by considering thirteen top professional qualities for problem forecasts with hypothetical results revealing appropriate effectiveness of the ready standard contrasted to various forecast solutions. On the contrary, Sonawane and Patil [10] offered a forecasting mechanism for coronary disease exploitation, multilayer perceptron semantic grid; the NN within a forecasted system accepts thirteen experimental choices as the input, as well as likewise, it learns taking advantage of the backpropagation formula to anticipate the incidence or lack of the heart problem in the individual with exactness of 98% for projection.

Dai et al. [11] suggested their job based on the case history schedule, and they have utilized benchmark dataset for finding out formulas notably support vector machine (SVM), AdaBoost, logistic regression (LR), and also naive Bayes (NB) classifiers in the direction of the forecast of cardiovascular disease with a precision of 82%. Vembandasamy et al. [12] utilized the NB formula for CVD recognition by evaluating the specifications.

The article "A Reliable Machine Intelligence Model for Accurate Identification of Cardiovascular Diseases Using Ensemble Techniques" was published in 2022. Journal: J Healthc Eng.

Radhimeenakshi [13] predicted a technique that achieved a mean precision of 86.43% for coronary cardiovascular disease recommended by utilizing the SVM even more as an artificial neural network (ANN), as well as offering a clinical option assistance framework for coronary health problem characterization.

Saqlain et al. [14], in their work, predicted distressing acknowledgment of falling short with variable details of individuals with coronary health problems using LR and random forest (RF) which achieved 80% and 60% accuracies. Fatima and Pasha [15] conferred a comparative evaluation of numerous algorithms as a study paper and displayed the home of ML formulas and tools for CVD analysis and prediction. Finally, Malav et al. [16] revealed their work to forecast the CVD utilizing *K*-means jumble and forecasted a crossbreed guideline on the UCI heart condition dataset by using choices from it.

Karaylan and Kilic [17] made use of the ANN classifier for the projection of the CVD by utilizing the back spreading formula for training the network and by utilizing thirteen expert choices as the input and preparing for the lack of exposure of cardiac-based maladies with an accuracy of 95%. Esfahani and Ghazanfari [18] anticipated an expert system technique on UCI Laboratory info, along with using expedition pattern solutions together with a decision tree (DT), NN, SVM, and NB, and authors achieved an accuracy of 86.8%.

An ANN model of a multilayer perceptron was presented, containing 18 neurons in the hidden layer. This model has a sensitivity of 89.4%, specificity of 57.4%, and accuracy of 82.5% in the testing group, and a sensitivity of 85.8%, specificity of 60.8%, and accuracy of 80.76% in the overall patients [19].

Shah et al. [20] presented crossbreed techniques that utilizes clinical examination results as the input and extracts a reduced dimensional feature established by utilizing the probabilistic principal component analysis (PPCA) classification of heart disease making use of the UCI dataset. Gavhane [21] made use of backbreeding multilayer perceptron (MLP) from calculation for predicting the presence of heart problems.

Sanketha Rathnayakc and Ganegoda [22] proposed a method to predict cardiovascular disease by proposing neural network classification. They also worked on showcasing risk levels of the person using models such as *K*-nearest neighbour (KNN), DT, and NB. Doppala et al. [23] presented a forecast model with various features with different combinations and a few known grouping strategies. The authors produced an upgraded performance level with an accuracy of 84.42% using the hybrid machine learning technique.

The article "A Reliable Machine Intelligence Model for Accurate Identification of Cardiovascular Diseases Using Ensemble Techniques" was published in 2022. Journal: J Healthc Eng.

Nasarian et al. [24] utilized the coronary artery disease (CAD) dataset, throughout which task area and environmental options, furthermore, to various clinical functions and results revealed that the anticipated quality option technique had generated the accuracy of 81.23% with SMOTE in addition to the XGBoost classifier. On the contrary, Alizadehsani et al. [25] utilized the growth of the Z-Alizadeh Sani dataset, having 54 characteristics with 303 subjects and all-brand new specific alternative collection standards. The authors proposed a novel feature selection algorithm. Meanwhile, the uncertainty in CAD prediction is tackled by discretizing the data.

Doppala et al. [26] prepared an ensemble system that recognized cardiac-based diseases with a precision of 85.24% that is much healthier when collated with existing AI strategies. Shankar et al. [27] applied a forecast design over real-life health center data. The authors used structured and disorganized person data to suggest a CNN policy as an illness threat prediction formula. The accuracy obtained utilizing the established model ranges between 85% and 88%.

Singh et al. [28] proposed an optimized CNN model using a MADE-based technique to optimize the COVID-19 condition. The model is created and executed to categorize the contaminated individuals. Experimental results show that the proposed model outperforms CNN, GA-based CNN, and PSO-based CNN models concerning the, *F*-measure, level of sensitivity, specificity, and kappa statistics which are1.2438%, 1.1378%, 1.3194%, and 1.1624%, respectively.

Bayu Adhi et al. [29] anticipated a method that beats any base classifiers within the set with relevance cross-validation of 10-fold. Our discovery design has performed more than the present existing versions that maintained old classifier sets and private classifiers regarding the accuracy of 93.55%. Doppala et al. [30] prepared a genetic crossbreed approach pattern loaded with an air precision pattern for different functional systems. The proposed model achieved an overall accuracy of 85.40% on 14 features. The projection accuracy inflated to 94.20% with nine functions where the energy of the forecasted system performed better on the function decrease.

Table 1 displays different models developed during the last decade and their achieved accuracies.

Singh et al. [31] suggested an ensemble deep discovering design for the COVID-19 category in upper body computed tomography (CT) scan pictures. The recommended set design used the three well-known models, particularly DCCNs, ResNet152V2, and VGG16. The recommended ensemble design has been tested on a big upper body CT dataset compared with fifteen affordable designs. Theoretical results disclose that the proposed set version exceeds the existing designs concerning the accuracy, *F*-measure, area under the curve (AUC), level of sensitivity, and specificity by 1.27%, 1.32%, 1.83%, 1.28%, and 1.83%, respectively.

The article "A Reliable Machine Intelligence Model for Accurate Identification of Cardiovascular Diseases Using Ensemble Techniques" was published in 2022. Journal: J Healthc Eng.

Kumar et al. [32] came up with a system that provides statistics to an android app. The evaluation has then executed a pretrained machine to know the model, and it is trained at the identical dataset deployed in firebase. Finally, LR is used for disease identification.

A. Akella and S. Akella [33] made a comparative study on 6 ML models and achieved the precision value above 80%, with the neural network model achieving precision above 93%. Finally, Waqas Nadeem et al. [34] presented a new architecture for cardiac disease prediction using the SVM. The proposed model has achieved 96.23% accuracy, which is significantly high compared to existing models.

Kumar et al. [32] discussed disease detection, and for the study, logistic regression is utilized for the forecast. Substantial experimental outcomes expose that the suggested version exceeds the competitive equipment finding out versions regarding precision and *F*-measure by 1.4765% and 1.2782, specifically, for the COVID-19 dataset. The recommended version surpasses the affordable device finding out versions in terms of precision and *F*-measure by 1.8274% and 1.7264, specifically, for the diabetes mellitus dataset.

Shorfuzzaman et al. [35] discussed a novel convolutional neural network- (CNN-) based deep learning blend structure employing the transfer learning idea. The proposed model accomplished an accuracy of 95.49%. Existing models' achieved accuracies are compared in Table 1.

## 3. Materials and Methods

The following section narrates the materials and methods used in this research work, including the proposed system architecture, experimental dataset description, data preprocessing, ML classifiers, proposed model algorithm, model accuracy computation, and performance evaluation metrics.

### 3.1. Proposed System Architecture

Three primary datasets on heart disease were collected for this study. Before performing the classification, data preprocessing has been performed. The main objective of performing this process is to avoid unwanted and missing values because they may impact the classifier's performance. So, providing hassle-free data to a classifier is more critical. The proposed ensemble model is a combination of naive Bayes, random forest, support vector machine, and XGBoost. The purpose of ensemble is to create multiple models and combine them to produce better results. A voting mechanism is used for classification towards the identification of heart disease.  Figure 1 demonstrates the proposed model architecture, and the consecutive sections narrate about working mechanisms at different stages present in the proposed architecture.

The article "A Reliable Machine Intelligence Model for Accurate Identification of Cardiovascular Diseases Using Ensemble Techniques" was published in 2022. Journal: J Healthc Eng.

### 3.2. Experimental Data Considered and Dataset Description

Three different datasets are used to carry out this research work:

1. Coronary disease dataset collected from the Cleveland repository [36] that consists of 303 subjects in total
2. A cumulative dataset of cardiovascular disease acquired from 5 different repositories that is not integrated before [37] consists of 1190 circumstances
3. The heart illness dataset was acquired from one of India's multispecialty hospitals [38], consisting of one thousand subjects

Because most clinical datasets are unbalanced, it is necessary to balance them for algorithms to perform better. When working with unbalanced datasets, selecting the appropriate assessment metric is crucial. In most cases, the *F*1 rating is all that is required as a metric. The *F*1 rating is a value between 0 and 1 that represents the harmonic suggestion of precision.

This section completely describes the features considered in this study in detail.  Table 2 displays the total number of features and their description.

Age: age is an essential chance element for developing CVD or coronary artery diseases.

Sex/gender: men are at extra danger of coronary heart ailment compared to ladies. As in most case studies, men will be addicted to hazardous habits such as tobacco and consumption of alcohol. Few prevalent diseases such as blood pressure and diabetes were common in both genders.

Angina: angina is a kind of pain in the chest where enough oxygen does not reach the chest muscles. It could sense pressure but can pass through different body parts such as the jaw, neck, arms, and shoulders.

Resting blood stress: high blood pressure can also be one of the main reasons for heart-based diseases. In addition, people having heavyweight issues, excessive cholesterol, and diabetes will be at a higher risk.

Serum cholesterol: an excessive stage of low-density lipoprotein cholesterol (“horrific” cholesterol) is most probable to narrow arteries. An excessive stage of triglycerides, a sort of blood fat related to a weight loss plan, additionally increases the chances of a heart assault. However, an excessive stage of high-density lipoprotein cholesterol (“exact” cholesterol) lowers your danger of a heart assault.

Fasting blood sugar: it is the condition of not generating sufficient hormones, and if blood sugar tries to rise based on these conditions, it in turn leads to a risk on the heart.

The article "A Reliable Machine Intelligence Model for Accurate Identification of Cardiovascular Diseases Using Ensemble Techniques" was published in 2022. Journal: J Healthc Eng.

Resting ECG: it is a test which measures the electrical heart activity. ECG can be used to detect different CVDs.

Max heart rate: due to excessive blood pressure, the acceleration rate of the heart will also increase. With excessive blood pressure, the rate may increase up to 10 beats per minute, and it can further increase, which may cause cardiac arrest.

Oldpeak: it is exercise-induced depression when compared to rest.

Target: datasets incorporate a characteristic named “target” to expose the analysis of coronary heart disorder in sufferers. In this state of affairs, zero indicates the disease absence, and 1 indicates the presence.

Three different datasets are used for this research, and respective heatmaps of the datasets are generated and represented in Figures 2–4. A heatmap is a two-dimensional visualization tool that helps describe the variable's intensity, pattern visualizations, and anomalies.

### 3.3. Data Preprocessing

Data generally contain noise, missing values, and unsuitable formats that cannot pass directly to machine learning models. Cleaning and preparing data for a machine learning model requires preprocessing, which improves the model's accuracy and efficiency. The accuracy of the details and the effectiveness of the classifier are dependent on how the features are handled. Because the dataset is linked to a minimax scalar, the features' values range from 0 to 1. If the losses in the value across a column or run are mathematical, the excellent worth will undoubtedly be attributed by the mean of the variable's entire conditions. If the feature is thought to have outliers, the mean can be altered using typical column value. The arrangement of the column can modify the impact on worth for a specific attribute [39].

### 3.4. Machine Learning Classifiers

This section deals with few benchmark machine learning algorithms and the proposed model.

#### 3.4.1. Support Vector Machine (SVM)

It divides information by tags. Bit method is used to match new information to finest from seasoned information to forecast unidentified target tag [29].

(1) $$\begin{array}{c} w^{T}\alpha +b=0, \end{array}$$

where *w*  is the dare dimensional coefficient vector and *b* is the offset value from the beginning. Option is acquired by presenting Lagrange multipliers in the direct instance and borders; sustain vectors are used as information factors.

(2) $$\begin{array}{c} w=\sum_{I=1}^{n}\alpha_{i}Y_{i}X_{i},\; \end{array}$$

where *n*  is the number of vectors and *Y*_*i*_  is the target tags to *X*.

The article "A Reliable Machine Intelligence Model for Accurate Identification of Cardiovascular Diseases Using Ensemble Techniques" was published in 2022. Journal: J Healthc Eng.

A straight discriminant function can be composed as

(3) $$\begin{array}{c} g\left(x\right)=sgn\left(\sum_{i=1}^{n}\alpha_{i}Y_{i}X_{i}^{T}X+b\right).\; \end{array}$$

The linear discriminant analysis provides a straight partition boundary between both recognized teams, bisecting the line between the centroids of the two groups. A discriminant plot tasks the data onto a solitary axis.

The kernel trick decision function is

(4) $$\begin{array}{c} g\left(x\right)=sgn\left(\sum_{i=1}^{n}\alpha_{i}Y_{i}K\left(\left(X_{i}+X\right)+b\right)\right).\; \end{array}$$

#### 3.4.2. Decision Tree (DT)

It consists of intertwining between indoor and outside nodes suggested for choice making and kid nodes for taking a look at complying with the node. Fallen leaf nodes have no child nodes and get in touch with the tag [29]. The basic structure of the decision tree is represented in Figure 5.

(5) $$\begin{array}{c} \text{Entropy}=\sum_{i=1}^{c}-P_{i}\log_{2}P_{i}.\; \end{array}$$

#### 3.4.3. Logistic Regression (LR)

It is mainly utilized for anticipating analysis. It reveals a direct partnership in between dependent (*y*) and independent (*x*) variables [30].

Sigmoid function:

(6) $$\begin{array}{c} h\theta \left(x\right)=g\theta^{T}-T, \end{array}$$

where *g*(*z*)=1/(1+*x*+*z*) and *h*(*x*)=1/(1+*x* − *z*).

LR cost function and logistic function are represented in Figure 6.

(7) $$\begin{array}{c} J\left(\theta \right)=\frac{1}{m}\sum_{i=1}^{m}\cos\;t\left(h\theta \left(x^{\left(i\right)}\right)y^{\left(i\right)}\right).\; \end{array}$$

#### 3.4.4. Naive Bayes

It is quite possibly the clearest, just as powerful classification equations. In like manner, this is utilized continuously because the NB classifier is an enthusiastic learner [29] represented in the following equation:

(8) $$\begin{array}{c} P\left(C|X\right)=\frac{P\left(X|C\right)P\left(C\right)}{P\left(X\right)},\; \end{array}$$

where *P*(*C|X*)  is the back chance, *P*(*X|C*)  is the likelihood, *P*(*C*)  is the class prior chance, and *P*(*X*)  is the predictor prior chance.

#### 3.4.5. Proposed Model

The voting classifier is one of the ensemble algorithm models. In the case of regression, the voting mechanism usually produces a prediction of the models' average. We have considered NB, RF, SVM, and gradient boosting classifiers for our study to build up the model, represented in Figure 1.

Every model version generates a forecast for each examination circumstance, with the most popular outcome forecast receiving the most votes. If none of the forecasts receives more than half of the votes, we can conclude that the set approach is unlikely to produce a consistent forecast in these conditions. Therefore, we predict the class $\;\hat{y\;}$ based on the popularity voting of every classifier *C*_*j*_ that is taken into consideration. (Figure 7).

(9) $$\begin{array}{c} \hat{y}=\text{mod }e\left\{C_{1}\left(x\right),C_{2}\left(x\right),\ldots ,C_{m}\left(x\right)\right\}. \end{array}$$

Majority voting is computed by associating weight *w*_*j*_ to the classifier *C*_*j*_.

(10) $$\begin{array}{c} \hat{y}=\underset{i}{\max}\sum_{j=1}^{m}w_{j}x_{A}\left(C_{j}\left(x\right)=i\right). \end{array}$$

*x*_*A*_ is the characteristic function *C*_*j*_(*x*)=*i*  ∈ *A*. *A* is a unique label set of a class.

The article "A Reliable Machine Intelligence Model for Accurate Identification of Cardiovascular Diseases Using Ensemble Techniques" was published in 2022. Journal: J Healthc Eng.

The predicted probability of the classifier is

(11) $$\begin{array}{c} \hat{y}=\underset{i}{\max}\sum_{j=1}^{m}w_{j}p_{ij}.\; \end{array}$$

The proposed algorithm is represented in Table 3.

## 4. Results and Discussion

In this research work, a strong voting classifier is identified to determine coronary sickness, tested on three different datasets. Each dataset has around 14 key features with different volumes of subjects. Datasets have been partitioned for both testing and training purposes, with a 60 : 40 split considered. This split also qualifies in such a manner that the underfitting problem is avoided when the fraction of testing data is smaller than the proportion of training data.

This research work is implemented on a machine with the following configuration and software: Python language is implemented on Jupyter Notebook 6.0.3 on Intel^®^ Core™ i7-4510U CPU@2.00 GHz 2.60 GHz, a 64 bit operating system with 8 GB RAM. Accuracies achieved with few benchmark algorithms on all the datasets used for this research work have been represented in Table 4.

Table 5 shows the proposed model performance with all the datasets used in the study.

On all datasets, the proposed model outperformed the current benchmark methods in terms of accuracy. In addition, results demonstrate that the generated model is reliable and can be used on any dataset, regardless of its size.  Table 6 shows the metrics of algorithms in terms of performance when compared to the suggested model.

### 4.1. Graphical Representation of Classifier Performance Metrics on Various Datasets

The graphs show a graphical summary of the findings obtained by several machine learning models and the suggested ensemble model and its performance measures. For instance, Figure 8 shows the performance of classifiers on the Cleveland dataset. In contrast, Figure 9 shows the performance of classifiers on the comprehensive dataset, and Figure 10 shows the performance of classifiers on the Mendeley dataset.

Heart disease datasets are subjected to several classification techniques. For example, on the Cleveland UCI repository dataset, our suggested model has an accuracy of 88.24%, 93.39% on the comprehensive dataset from IEEE DataPort, and 96.75% on the cardiovascular disease dataset, Mendeley Data Centre.

The article "A Reliable Machine Intelligence Model for Accurate Identification of Cardiovascular Diseases Using Ensemble Techniques" was published in 2022. Journal: J Healthc Eng.

### 4.2. AUC and ROC Representations

Measuring performance is a crucial task. As a result, we can forecast an AUC-ROC contour once it incorporates a categorization issue. It is one of the most important criteria for assessing the efficiency of any form of category model.

Figures 11–13 show the generated ROC curves for all of the models on the datasets utilized in this study. The figures provide a better understanding of the proposed model's performance when compared with benchmark algorithms.

## 5. Conclusion

As shown in Table 4, a trustworthy ensemble strategy advocated in this research work outperformed seven benchmark algorithms effectively. Our proposed model produced more accurate results of 96.75% on the cardiovascular disease dataset obtained from the Mendeley Data Center, 93.39% on the comprehensive dataset obtained from IEEE DataPort, and 88.24% on the Cleveland dataset obtained from the UCI repository, according to extensive experimental results. Compared to the existing models on all three datasets utilized in the study, the suggested model is more accurate and yields higher values. As shown in Table 5, the proposed model is consistent in delivering more accurate results across various datasets, saving patients' and healthcare professionals' time in decision-making.

## Figures and Tables

**Figure 1:** Proposed model architecture.

**Figure 2:** Heatmap of the heart disease dataset obtained from the Cleveland repository.

**Figure 3:** Heatmap of the dataset obtained from IEEE DataPort.

**Figure 4:** Heatmap of the cardiovascular disease dataset obtained from the Mendeley Data Center.

**Figure 5:** Representation of the decision tree [40].

**Figure 6:** Representation of the logistic function [41].

**Figure 7:** Representation of naive Bayes [38].

**Figure 8:** Classifiers' performance on the Cleveland dataset.

**Figure 9:** Classifiers' performance on the comprehensive dataset.

**Figure 10:** Classifiers' performance on the Mendeley dataset.

**Figure 11:** ROC curve for all models on the Cleveland dataset.

**Figure 12:** ROC curve for all models on the comprehensive dataset.

**Figure 13:** ROC curve for all models on the Mendeley dataset.

**Table 1:** Existing models' accuracy comparison.

Authors	Model used	Accuracy (%)
AI-Milli [9]	NN	81
Sonawane and Patil [10]	MPNN	98
Dai et al. [11]	AdaBoost	82
Radhimeenakshi [13]	SVM, ANN	86
Saqlain et al. [14]	LR and RF	80.69
Karaylan and Kilic [17]	ANN	95
Esfahani and Ghazanfari [18]	DT	86.80
Cheng and Chiu [19]	ANN	82.5
Doppala et al. [23]	Hybrid model	84.40
Nasarian et al. [24]	Hybrid feature selection	81.23
Doppala et al. [26]	Ensemble	85.24
Kumar et al. [32]	CNN	88
Bayu Adhi et al. [29]	Ensemble	93.55
Doppala et al. [30]	GA-RBF	85.40, 94.20
Waqas Nadeem et al. [34]	SVM	96.23

The article "A Reliable Machine Intelligence Model for Accurate Identification of Cardiovascular Diseases Using Ensemble Techniques" was published in 2022. Journal: J Healthc Eng.

**Table 2:** Dataset attributes' description [33].

S. no.	Cleveland dataset features	Comprehensive dataset features	Mendeley dataset features	Unit
1	Age	Age	Age	In years
2	Sex	Sex	Gender	1, 0 (0 = female; 1 = male)
3	cp	Chest pain type	Chest pain	Value 0: typical angina; value 1: atypical angina
4	trestbps	Resting bps	Resting BP	94–200 (in mmHg)
5	chol	Cholesterol	Serum cholesterol	126–564 (in mg/dl)
6	fbs	Fasting blood sugar	Fasting blood sugar	0, 1 > 120 mg/dl (0 = false; 1 = true)
7	restecg	Resting ECG	Restingrelectro	0, 1, 2 (value 0: normal; value 1: having ST-T-wave abnormality (T-wave inversions and/or ST elevation or depression of >0.05 mV); value 2: showing probable or definite left ventricular hypertrophy by Estes criteria
8	thalach	Max heart rate	Max heart rate	71–202
9	exang	Exercise angina	Exercise angina	0, 1 (0 = no; 1 = yes)
10	Oldpeak	Oldpeak	Oldpeak	0–6.2
11	Slope	ST slope	Slope	1, 2, 3 (1-upsloping, 2-flat, and 3-downsloping)
12	ca	—	No. of major vessels	0, 1, 2, 3
13	thal	—	—	Thalassemia display, 3 = normal, 6 = fixed, and 7 = reversible defect
14	Target	Target	Target	0, 1 (0 = absence of heart disease; 1 = presence of heart disease)

**Table 3:** Proposed algorithm.

Algorithm
**Procedure ** *LOAD (heart_disease_data)*
**Procedure ** *DATA_SPLIT (heart_disease_data)*
Train_data, Test_data = split (heart_disease_data,lables)
**return** Train_data, Test_data
*voting*=”*soft*”
*C1= Naive_Bayes (Training_data, Train_label, Testing_data)*
*C2= Random_Forest (Training_data, Train_label, Testing_data)*
*C3=Support_Vector_Machine (Training_data, Train_label, Testing_data)*
*C4= Gradient_Boosting (Training_data, Train_label, Testing_data)*
**Procedure ** *ENSEMBLE_MODEL (Train_data, Train_label, Test_data)*
*soft_voting_classifier=concatenate (C1,C2,C3,C4)*
*soft_voting_classifier.fit (Train_data, Train_label)*
*predictions=soft_voting_classifier.predict(Testing_data)*

**Table 4:** Achieved accuracies using benchmark classifiers.

Classification technique	Accuracy (%) achieved with the Cleveland dataset	Accuracy (%) achieved with the comprehensive dataset	Accuracy (%) achieved with the Mendeley dataset
Decision tree	77.86	82.56	95
Random forest	78.68	90.75	95.12
Naive Bayes	81.14	84.24	94.25
Logistic regression	81.96	84.03	95.25
Support vector machine	79.05	81.52	93.15
Gradient boosting	81.14	86.13	95.15
XGBoost	80.32	88.23	96.12

The article "A Reliable Machine Intelligence Model for Accurate Identification of Cardiovascular Diseases Using Ensemble Techniques" was published in 2022. Journal: J Healthc Eng.

**Table 5:** Proposed model performance representation.

Classification technique	Accuracy (%) achieved with the Cleveland dataset	Accuracy (%) achieved with the comprehensive dataset	Accuracy (%) achieved with the Mendeley dataset
Proposed ensemble model	88.24	93.39	96.75

**Table 6:** Performance metrics of all the machine learning models.

Classification technique	Accuracy (%) achieved with the Cleveland dataset	Sensitivity	Specificity	Precision	Recall	*F*1-score	MCC
Decision tree	77.86	0.81	0.73	0.77	0.81	0.79	0.55
Random forest	78.68	0.78	0.77	0.80	0.78	0.79	0.55
Naive Bayes	81.14	0.87	0.73	0.79	0.87	0.83	0.62
Logistic regression	81.96	0.93	0.66	0.76	0.790.	0.84	0.63
Support vector machine	79.05	0.77	0.75	0.79	0.85	0.78	0.54
Gradient boosting	81.14	0.93	0.66	0.76	0.93	0.84	0.63
XGBoost	80.32	0.87	0.71	0.78	0.87	0.82	0.60
Proposed ensemble model	88.24	0.91	0.84	0.85	0.90	0.88	0.76

Classification technique	Accuracy (%) achieved with the comprehensive dataset	Sensitivity	Specificity	Precision	Recall	*F*1-score	MCC

Decision tree	82.56	0.79	0.85	0.83	0.79	0.81	0.65
Random forest	90.75	0.93	0.88	0.88	0.93	0.90	0.81
Naive Bayes	84.24	0.85	0.82	0.82	0.85	0.84	0.68
Logistic regression	84.03	0.87	0.80	0.81	0.87	0.84	0.68
Support vector machine	81.52	0.83	0.82	0.82	0.84	0.83	0.69
Gradient boosting	86.13	0.92	0.79	0.81	0.92	0.86	0.72
XGBoost	83.23	0.91	0.84	0.85	0.91	0.88	0.76
Proposed ensemble model	93.39	0.94	0.89	0.99	0.88	0.90	0.85

Classification technique	Accuracy (%) achieved with the Mendeley dataset	Sensitivity	Specificity	Precision	Recall	*F*1-score	MCC

Decision tree	95	0.95	0.94	0.96	0.95	0.95	0.88
Random forest	95.12	0.94	0.96	0.97	0.94	0.96	0.90
Naive Bayes	94.25	0.95	0.90	0.94	0.95	0.94	0.86
Logistic regression	95.25	0.97	0.95	0.97	0.97	0.97	0.92
Support vector machine	93.15	0.95	0.90	0.93	0.95	0.93	0.85
Gradient boosting	95.15	0.95	0.95	0.97	0.95	0.96	0.90
XGBoost	96.12	0.96	0.95	0.97	0.96	0.96	0.92
Proposed ensemble model	96.75	0.96	0.97	0.98	0.96	0.97	0.93

## Data Availability

The data used to support the findings of this study are available from the corresponding author upon request.
